The article "Knockdown of TRIM65 inhibits lung cancer cell proliferation, migration and invasion: A therapeutic target in human lung cancer" was retracted in 2024. Reason: duplicated images.

# Knockdown of TRIM65 inhibits lung cancer cell proliferation, migration and invasion: A therapeutic target in human lung cancer

**DOI:** 10.18632/oncotarget.13131

**Published:** 2016-11-05

**Authors:** Xiao-Lin Wang, Wei-Ping Shi, Hong-Can Shi, Shi-Chun Lu, Kang Wang, Chao Sun, Jian-Sheng He, Wei-Guo Jin, Xiao-Xia Lv, Hui Zou, Yu-Sheng Shu

**Affiliations:** ^1^ Department of Thoracic Surgery, Northern Jiangsu People's Hospital and Clinical Medical College of Yangzhou University, Yangzhou 225001, People's Republic of China

**Keywords:** lung cancer, TRIM65, apoptosis, migration

## Abstract

Lung cancer is the most commonly diagnosed type of cancer worldwide. Although TRIM65 is an important protein involved in white matter lesion, the role of TRIM65 in human cancer remains less understood. Here, we reported that TRIM65 was significantly overexpressed in lung cancer tissues compared with adjacent normal lung tissues. Furthermore, TRIM65 expression was closely related to overall survival of patients with lung cancer. Knock down of TRIM65 in two lung cancer cell lines, SPC-A-1 and NCI-H358, resulted in a significant reduction in cell proliferation, migration, invasion and adhesion and a dramatic increase in G0-G1 phase arrest and apoptosis. *In vivo* tumorigenesis experiment also revealed that depletion of TRIM65 expression inhibited NCI-H358 cell growth. Moreover, based on gene set enrichment analysis (GSEA) with The Cancer Genome Atlas (TCGA) dataset, we found that TRIM65 was positive related to cell cycle, metastasis up and RHOA-REG pathways, which was further validated by RT-PCR and Western blot in TRIM65 knockdown lung cancer cells and indicated a possible mechanism underlying its effects on lung cancer. In summary, our study suggests that TRIM65 may work as an oncogene and a new effective therapeutic target for lung cancer treatment.

## INTRODUCTION

Malignant tumor cells use their inherent ability of migration, invasion of adjacent tissue and blood vessels, and finally to metastasize [1]. Metastasis, the most critical prognostic factor, is composed of multiple steps as follows: attachment of tumor cells to the extracellular matrix (ECM), secretion of matrix-degrading enzymes, migration of tumor cells through the degraded matrix, invasion of blood vessels and circulation, and implantation into other distant organs [2]. Cell migration is a multistep process responded to migration and chemotaxis stimulation, which is initiated by the formation of membrane protrusions [3]. Therefore, understanding the underlying mechanisms of cell migration is necessary for our understanding of the development and progression of the disease.

Lung cancer is a common type of cancer worldwide and more than 75% of all lung cancers consist of non-small cell lung carcinoma (NSCLC) [4]. Although radiation therapy has been established as a standard treatment for lung cancer and has improved survival of the patients [5], the major health threat for lung cancer is death due to metastasis. For developing more effective therapies, a better understanding of the molecular biology of lung cancer is important to obtain.

The article "Knockdown of TRIM65 inhibits lung cancer cell proliferation, migration and invasion: A therapeutic target in human lung cancer" was retracted in 2024. Reason: duplicated images.

Gene change is a marker of human cancer. In recent years, the field of cancer genomics has made remarkable progress in determining the genetic disease of cancer. TRIM65 belongs to the TRIM (tripartite motif-containing protein) family has been identified as an ubiquitin ligase (E3) and possesses critical functions in a variety of cellular processes [6]. TRIM65 was widely expressed in human lung cancer tissues and inactivates p53 through mediating p53 ubiquitination and degradation [7]. However, there have been no reports on possible mechanism of TRIM65 associates with lung cancer carcinogenesis.

In this study, we demonstrated that up-regulation of TRIM65 is closely related to human lung cancer tumorigenesis, and knockdown of TRIM65 reduces the cell growth, invasion, migration and adhesion, and arrests cell cycle and promotes apoptosis of human lung cancer cells. Furthermore, gene set enrichment analysis (GSEA) using The Cancer Genome Atlas (TCGA) dataset showed that TRIM65 was positive related with cell cycle, metastasis up and RHOA-REG pathways, which was further validated in human lung cancer cells with TRIM65 knockdown. Our data provide new insights into the molecular function of TRIM65 as well as its regulatory mechanisms in lung cancer.

## RESULTS

### TRIM65 upregulation in human lung cancer tissues and cell lines

TRIM65 expression was marked overexpression in human lung cancer tissues when in comparison with the adjacent normal lung tissues of patients from TCGA dataset (Figure 1A) and Northern Jiangsu People's Hospital independent dataset (Figure 1B). Next, we examined the relationship between TRIM65 expression and clinicopathological features of the lung cancer patients from GEO dataset (Access id: GSE50081). We detected the expression level of TRIM65 of 177 lung cancer patients' tissues divided into two group using TRIM65 median value (median value=3.451). Chi-square test indicated that the higher TRIM65 expression correlated with the poor prognosis (Figure 1C). However, TRIM65 expression was not correlated with gender, age, tumor histology and clinical stage (data not shown).

**Figure 1:** TRIM65 expression in human lung cancer tissues and cell lines **A.** TRIM65 mRNA level was significantly higher in human lung cancer tissues (n = 488) than in adjacent-normal lung tissues (n = 58) from the TCGA dataset. **B**, **E.** TRIM65 mRNA and protein levels were significantly increased in human lung cancer tissues (n = 40) compared with adjacent-normal lung tissues of patients (n = 40) from patients admitted to Hospital from 2009 to 2010. T: tumor tissue; N: adjacent-normal lung tissue. **C.** The overall survival time of 177 patients with lung cancer. **D.** Expression of TRIM65 was determined by immunohistochemistry staining in human lung cancer tissues. Scale bars: 100 μm. **F.** TRIM65 expression level in five human cancer cell lines was analyzed by RT-PCR and Western blot. ***P < 0.01 compared with adjacent normal lung cancer tissues.

The article "Knockdown of TRIM65 inhibits lung cancer cell proliferation, migration and invasion: A therapeutic target in human lung cancer" was retracted in 2024. Reason: duplicated images.

To assess the protein levels of TRIM65 in lung cancer tissues, immunohistochemistry (IHC) staining of TRIM65 was performed in 40 human lung cancer specimens. As shown in Figure 1D, tumor tissues showed high expression compared with that in adjacent normal lung cancer tissues. TRIM65 protein expression results were similarly observed in randomly selected four paired lung cancer and adjacent normal tissues measured by Western blot analysis (Figure 1E).

Having documented upregulation of TRIM65 associates with poor prognosis of lung cancer patients, we further investigated the effect of TRIM65 on lung cancer tumorigenesis both *in vitro* and *in vivo*. We first examined the expression levels of TRIM65 in five lung cancer cell lines, A549, SPC-A-1, NCI-H358, NCI-H1975, HCI-H446 and HCI-H292 by RT-PCR and Western blot (Figure 1F). The highest expression of TRIM65 was detected in SPC-A-1 and NCI-H358 cell lines in comparison with the other cell lines, while TRIM65 was expressed in lower level in NCI-H1975 and NCI-H446 cells.

### Knockdown of TRIM65 inhibits cell proliferation of lung cancer cells *in vitro*

In order to knockdown TRIM65, we also transfected siRNA targeted human TRIM65 mRNA (siRNA-TRIM65) into SPC-A-1 and NCI-H358 cells. The efficacy of TRIM65 knockdown was examined by RT-PCR and Western blot. Meanwhile, a scramble siRNA was used as a negative control (siRNA-NC). Figure 2A and 2B showed that the mRNA and protein levels of TRIM65 were markedly decreased in SPC-A-1 and NCI-H358 cells after transfected with siRNA-TRIM65.

**Figure 2:** Knockdown of TRIM65 inhibits cell proliferation of human lung cancer cell lines Knockdown of TRIM65 by siRNA showed notably expression inhibited in mRNA and protein levels in **A.** SPC-A-1 and **B.** NCI-H358 cells. Cell proliferation was detected in siRNA-NC or siRNA-TRIM65 transfected **C.** SPC-A-1 and **D.** NCI-H358 cells by CCK-8 assay. ***P<0.001 compared with siRNA-NC group. NC: negative control.

The article "Knockdown of TRIM65 inhibits lung cancer cell proliferation, migration and invasion: A therapeutic target in human lung cancer" was retracted in 2024. Reason: duplicated images.

Next, we determined whether TRIM65 knockdown affects the lung cancer cell proliferation at progressive stages of tumorigenesis. Towards this end, cellular proliferation was determined using CCK-8 assay. We noted that TRIM65 knockdown remarkably inhibited the proliferation of SPC-A-1 and NCI-H358 cells after 48 h and 72 h (Figure 2C and 2D).

### Knockdown of TRIM65 induces cell cycle arrest and apoptosis in lung cancer cells

To further investigate the role of TRIM65 in lung cancer cell proliferation, cell cycle was analyzed in SPC-A-1 and NCI-H358 cells. Our results demonstrated that downregulation of TRIM65 significantly decreased the rate of S and G2-M phase cells and increased the rate of G0-G1 phase cells in both cell lines (Figure 3A and 3B). Then, Annexin V-FITC/PI staining assay was performed to evaluate the role of TRIM65 in cell apoptosis in SPC-A-1 and NCI-H358 cells. As shown in Figure 3C-3F, downregulation of TRIM65 in SPC-A-1 and NCI-H358 cells markedly increased cell apoptotic rates in comparison with siRNA-NC.

**Figure 3:** Knockdown of TRIM65 inhibits cell cycle progression and induces apoptosis of human lung cancer cell lines SPC-A-1 and NCI-H358cells were transfected with siRNA-NC or siRNA-TRIM65 and collected 48 h later cells. Cell cycle profile was analyzed using flow cytometry in **A.** SPC-A-1 and **B.** NCI-H358 cells. **C**, **E.** SPC-A-1 and **D**, **F.** NCI-H358 cell apoptosis was analyzed by Annexin V/PI staining. *P<0.05, **P<0. 01, ***P<0.001 compared with siRNA-NC group. NC: negative control.

### Knockdown of TRIM65 inhibits migration, invasion and adhesion in lung cancer cells

Evidences have shown that inhibition of cell-cell and/or cell-matrix adhesive function correlates with tumor migration and invasion. After 48 h of incubation, compared with the siRNA-NC cells, both SPC-A-1 and NCI-H358 cells (Figure 4A, 4D and 4E) showed significantly decreased migratory ability. Using a matrigel-coated transwell chamber, we found that siRNA-TRIM65 transfected into SPC-A-1 and NCI-H358 cells significantly reduced the invasive capacity compared with the corresponding siRNA-NC groups (Figure 4B, 4F and 4G). Furthermore, we also detect the adhesive capacity of SPC-A-1 and NCI-H358 cells with siRNA-TRIM65 transfection. The results observed that TRIM65 knockdown notably repressed the SPC-A-1 and NCI-H358 cells adhesive ability compared with the corresponding siRNA-NC groups (Figure 4C, 4H and 4I). Our results demonstrated a function of TRIM65 in promoting lung cancer cell migration, invasion and adhesion.

**Figure 4:** Knockdown of TRIM65 inhibits migration, invasion and adhesion in human lung cancer cell lines SPC-A-1 and NCI-H358 cells were transfected with siRNA-NC or siRNA-TRIM65. **A**, **D**, **E.** Cell migration, **B**, **F**, **G.** invasion and **C**, **H**, **I.** adhesion assay were performed. ***P<0.001 compared with siRNA-NC group. NC: negative control. Scale bars: 100 μm.

The article "Knockdown of TRIM65 inhibits lung cancer cell proliferation, migration and invasion: A therapeutic target in human lung cancer" was retracted in 2024. Reason: duplicated images.

### Effect of TRIM65 knockdown on apoptosis- and migration-related protein expressions

Then, three core proteins involved in the apoptosis, inducing Bcl-2, Bax and caspase-3, and four core proteins involved in migration, including Twist1, MMP-2, MMP-9 and E-cadherin, were predicted to be TRIM65 targets. To experimentally validate TRIM65 regulation of these genes, we detected the mRNA and protein levels of the target genes by RT-PCR and Western blot. As shown in Figure 5A-5D, the mRNA levels of Bcl-2, Twist1, MMP-2 and MMP-9 in SPC-A-1 and NCI-H358 cells were markedly decreased by siRNA-TRIM65, compared with siRNA-NC groups, while the mRNA levels of Bax, caspse-3 and E-cadherin were remarkably increased. The similar results were also found in protein levels of these genes in SPC-A-1 and NCI-H358 cells (Figure 5E and 5F).

**Figure 5:** Effect of TRIM65 knockdown on the expression of proteins correlated with apoptosis and migration SPC-A-1 and NCI-H358 cells were transfected with siRNA-NC or siRNA-TRIM65. RT-PCR and Western blot analysis identified significant increase in Bax, caspase-3 and E-cadherin, while decrease in Bcl-2, Twist1, MMP-2 and MMP-9 expression in **A**, **B**, **E.** SPC-A-1 and **C**, **D**, **F.** NCI-H358 cells infected with siRNA-TRIM65. ***P<0.001 compared with siRNA-NC group. NC: negative control.

### Identification of TRIM65-associated biological pathways by GSEA

To assess the TRIM65-related pathways on an unbiased basis, we performed GSEA using data from the TCGA cohort. The expression level of TRIM65 gene was used as the phenotype label. As shown in Figure 6A, cell cycle, metastasis up and RHOA-REG pathways were identified to be significantly associated with TRIM65 expression in the TCGA cohort.

**Figure 6:** Mechanisms of TRIM65 exert their functions in human lung cancer cell lines GSEA compared TRIM65 higher expression group (red) against TRIM65 lower expression group (blue) of lung cancer patients in the TCGA dataset. Enrichment plots are shown for a set of activated genes related to **A.** cell cycle, **B.** metastasis up and **C.** RHOA-REG pathways. RT-PCR and Western blot analysis identified significant decrease in PCNA, Cyclin D1, CDC25A, KPNA2, MELK, KIF2C, RHOA, ROCK1 and ARHGAP5, while increase in DLC1 expression in B, C. U251 and **D**, **E.** T98G cells infected with pLVTHM-HDAC1-shRNA. ***P<0.001 compared with siRNA-NC group. NC: negative control.

The article "Knockdown of TRIM65 inhibits lung cancer cell proliferation, migration and invasion: A therapeutic target in human lung cancer" was retracted in 2024. Reason: duplicated images.

To validate the GSEA analysis of TRIM65, we analyzed the mRNA and protein levels of the cell cycle, metastasis up and RHOA-REG pathways related factors in siRNA-TRIM65 transfected SPC-A-1 and NCI-H358 cells. As shown in Figure 6B and 6C, the mRNA and protein levels of cell cycle-related factors [Proliferating cell nuclear antigen (PCNA), Cyclin D1 and Cell division cycle 25A (CDC25A)], metastasis up-related factor [Karyopherin Subunit Alpha 2 (KPNA2), Maternal Embryonic Leucine Zipper Kinase (MELK) and Kinesin Family Member 2C (KIF2C)] and RHOA-REG-related factor [Ras Homolog Family Member A (RHOA), Rho Associated Coiled-Coil Containing Protein Kinase 1 (ROCK1) and Rho GTPase Activating Protein 5 (ARHGAP5)] were significantly lower in siRNA-TRIM65 transfected SPC-A-1 cells than in corresponding siRNA-NC cells, while the RHOA-REG-related factor (Deleted in liver cancer 1, DLC1) was remarkably higher in siRNA-TRIM65 transfected SPC-A-1 cells. Consistent with functional characterization measured in SPC-A-1 cells, both NCI-H358 cells displayed the similar results (Figure 6D and 6E).

### Downregulation of TRIM65 suppresses tumor growth of lung cancer cells *in vivo*

Then, we wonder whether knockdown of TRIM65 cells could also inhibit tumor growth in lung cancer *in vivo*. After 45 days, the TRIM65 expression in mice with NCI-H358 cells transfected with siRNA-TRIM65 was significant decrease compared to the siRNA-NC mice (Figure 7A). Compared with siRNA-NC group, a significant decrease of Ki67-positive cells and a notable increase of apoptotic cells were observed in tumors formed from knockdown TRIM65 cells by immunohistochemistry assay and TUNEL (Figure 7B). Moreover, siRNA-TRIM65-treated tumors grew much slower than the siRNA-NC-treated tumors in mice (Figure 7C). 45 days after inoculation the mice were killed and the average tumor weights of siRNA-NC and siRNA-TRIM65 mice were 3.91 ± 0.51 g and 1.35 ± 0.53 g, respectively (Figure 7D). Additionally, we also determined the expression of cell cycle and metastasis-related proteins *in vivo*. As shown in Figure 7E, the expression of all the proteins was decreased except E-cadherin in mice *in vivo* with siRNA-NC treated. These data suggest that siRNA-TRIM65 had similar effects *in vitro* and *in vivo*.

**Figure 7:** Knockdown of TRIM65 in human lung cancer cells reduces tumor growth *in vivo* NCI-H358 cells infected with siRNA-NC or siRNA-TRIM65 were subcutaneously injected in armpit of nude mice. **A.** TRIM65 expression was measured by Western blot; **B.** Ki67 expression and apoptosis were detected by immunohistochemistry andTUNEL assays. Scale bars: 100 μm. **C.** Tumor volume and **D.** weight were also measured after TRIM65 knockdown. **E.** Expression of cell cycle and metastasis-related proteins was measured by Western blot assay *in vivo*. ***P<0.001 compared with siRNA-NC group. NC: negative control.

The article "Knockdown of TRIM65 inhibits lung cancer cell proliferation, migration and invasion: A therapeutic target in human lung cancer" was retracted in 2024. Reason: duplicated images.

### Association of TRIM65 with RhoA

To elucidate the underlying mechanisms by which TRIM65 exerts its function in lung cancer pathogenesis, we identified protein candidates that functionally associated with TRIM65. As shown in Figure 8A, we explored the nature of the interaction between TRIM65 and RhoA by using Co-immunoprecipitiation in NCI-H358 cells. The result obtained from the Co-immunoprecipitiation experiments indicated that RhoA directly interacts with TRIM65.

**Figure 8:** TRIM65 binds to RhoA *in vitro* **A.** Co-immunoprecipitation showed that TRIM65 interacts with RhoA in the NCI-H358 cells. **B.** The expression of p-ERK1/2, ERK1/2, p-JNK1/2 and JNK1/2 was measured by Western blot assay.

As RhoA directly interacted with TRIM65, we wonder whether RhoA associated with the lung cancer tumorigenesis. We thus introduced RhoA inhibitor, exoenzyme C3 transferase, in siRNA-TRIM65 transfected or pLV-IRES-eGFP-TRIM65 infected NCI-H1975 cells. As shown in Figure 8B, the expression of p-ERK1/2 and p-JNK1/2 was significantly decreased in siRNA-TRIM65 and exoenzyme C3 transferase treated cells, while pLV-IRES-eGFP-TRIM65 alone or combined with exoenzyme C3 transferase treatment showed increased expression of p-ERK1/2 and p-JNK1/2, compared with untreated NCI-H1975 cells. However, the expression of ERK1/2 and JNK1/2 was not changed in each group.

## DISCUSSION

TRIM65 is a member of the tripartite motif family responsible for regulation of miRNA processing. Although the distribution and function of TRIM65 are unknown, Li et al. cloned a TRIM65 isoform which lacks exon 5 from the T98 glioblastoma cell line [8]. In this study, we observed that TRIM65 expression was increased in lung cancer tissues compared with adjacent normal lung tissues, which was supported by lung cancer patients' data from TCGA. Moreover, TRIM65 expression was associated with patients' survival rate. These data indicated the prognostic value of TRIM65 in lung cancer.

Our findings showed that knockdown of TRIM65 remarkably inhibited cell proliferation, migration, invasion and adhesion of lung cancer cells, while overexpression of TRIM65 promoted cell proliferation and motility in lung cancer cell line, NCI-H1975 (Figure S1). Thus, the increased expression of TRIM65 may be correlated with the increased cell proliferation, invasion and migration of lung cancer.

In the present study, three core proteins involved in the apoptosis, inducing Bcl-2, Bax and caspase-3, and four core proteins involved in migration, including Twist1, MMP-2, MMP-9 and E-cadherin, were predicted to be TRIM65 targets. The functional loss of Bax protein may play an important role in the development and progression of many types of cancer [9, 10]. The inhibition of apoptosis appears to occur through the down-regulation of Bax and caspase-3 in lung cancer cells, which thereby prevent apoptotic cascades [11, 12]. Consistent with the previous studies, Twist1 dramatically promoted cell migration in lung cancer cells [13]. Moreover, Huang et al. evidenced that up-regulation of MMP2 and MMP9 is one of the mechanisms by which Skp2 promotes cell invasion in lung cancer cells [14], suggesting an important role of MMP2 and MMP9 in tumor metastasis.

The article "Knockdown of TRIM65 inhibits lung cancer cell proliferation, migration and invasion: A therapeutic target in human lung cancer" was retracted in 2024. Reason: duplicated images.

The exact pathway that TRIM65 may regulate in lung cancer remains unclear. Our GSEA results indicated that TRIM65 was positively correlated with cell cycle, metastasis up and RHOA-REG pathways. We observed that the expression of cell cycle-related factors (PCNA, CyclinD1 and CDC25A), the expression of metastasis up-related factors (KPNA2, MELK and KIF2C) and RHOA-REG pathway-related factors (RHOA, ROCK1 and ARHGAP5) was lower, while DLC1 was higher in lung cancer cells with TRIM65 knockdown. Decreased PCNA expression in lung cancer showed inhibitory effects of tumor cell proliferation and cell cycle [15]. Wang et al. has reported that PCNA may play an important role in the development of NSCLC in VEGFA regulatory network, as a potential molecular marker for lung cancer [16]. CDC25A inactivation is a critical rate-limiting step of carcinogenesis and plays an important role in DNA damage-induced S-G2 checkpoint [17]. Moreover, it has been shown that artificial induction of CyclinD1 mRNA expression in breast cancer cells mimics estrogen effects and is sufficient to drive S-phase entry [18]. The abnormal expression of KPNA2 indicates a poor prognosis and correlated with the malignant transformation of cancer cells [19]. Inhibition of MELK obviously inhibited cell proliferation and migration of prostate cancer cells, and may be a new way of treating cancer patients with high-risk subgroups [20]. MicroRNA-148a suppresses epithelial-to-mesenchymal transition (EMT) by targeting ROCK1 in NSCLC cells, suggesting an important role of ROCK1 in EMT [21]. miR-486-5p downregulation promotes cell proliferation, migration and invasion *in vitro* and metastasis in mice by reduced expression of ARHGAP5 in lung cancer [22]. However, Healy et al. reported that ectopic DLC-1 expression dramatically reduces proliferation and tumorigenicity of NSCLC cells [23].

Recent studies have demonstrated TRIM65 interacts with TNRC6 in HEK 293 cells and regulates TNRC6 ubiquitination and stability [24]. TRIM65 up-regulation enhanced tumor growth and knockdown of TRIM65 displays opposite effect in NSCLC cells, mechanistically through binding to p53, one of the most critical tumor suppressor [25]. In this study, we revealed that TRIM65 directly bound to RhoA in NCI-358 cells, suggesting that implicate signaling through RhoA pathway as a critical downstream mechanism by which TRIM65 may regulate changes in the cell growth, cell cycle, apoptosis and motility. Induction of exogenous expression of ANLN enhanced the migrating ability of NSCLC cells by interacting with RhoA [26]. Furthermore, the activated ERK1/2 and JNK1/2 were also found in NCI-H1975 cells after pLV-IRES-eGFP-TRIM65 transfection and treatment of exoenzyme C3 transferase, a RhoA inhibitor widely used. However, TRIM65 knockdown inactivated ERK1/2 and JNK1/2 signaling. In agreement with our findings, Tang et al. showed that ERK and JNK pathways involved in MMP9 upregulation-induced lung cancer cell invasion [27].

The article "Knockdown of TRIM65 inhibits lung cancer cell proliferation, migration and invasion: A therapeutic target in human lung cancer" was retracted in 2024. Reason: duplicated images.

In conclusion, our study indicated that TRIM65 expression is remarkably up-regulated in lung cancer tissues. Depletion of TRIM65 is able to suppress lung cancer cell proliferation, migration, invasion and adhesion by cell cycle, metastasis up and RHOA-REG pathway. Therefore, TRIM65 may be regarded as an oncogene with important value for lung cancer patients as an unfavorable progression indicator, and can be used as a therapeutic target in the future.

## MATERIALS AND METHODS

### Cell culture and human lung cancer tissues collection

The human lung cancer cell lines, A549, SPC-A-1, NCI-H358, NCI-H1975, HCI-H446 and HCI-H292 cells were from the American Type Culture Collection (ATCC, Rockville, MD, USA). All cells were cultured in RMPI-1640 (Hyclone, Logan, UT, USA) supplemented with 10% fetal bovine serum (Hyclone) and 1% penicillin-streptomycin solution (Gibco). Cells were cultured at 37°C in an atmosphere of 5% CO_2_.

40 pairs of lung cancer tissues and adjacent normal lung tissues was obtained from patients who underwent surgery at Northern Jiangsu People's Hospital and Clinical Medical College of Yangzhou University from Feb 2011 to May 2015. The study protocol was approved by the ethics committee of Northern Jiangsu People's Hospital and Clinical Medical College of Yangzhou University. Written informed consents were obtained from all participants in this study. All the research was carried out in accordance with the provisions of the Helsinki Declaration of 1975.

### Immunohistochemistry

Tissue sections were cut and mounted on slides. After de-waxing and rehydration, the sections were antigen-retrieved in 10 mm citrate buffer for 5 min at 100°C. Endogenous peroxidase activity and non-specific antigens were blocked with 3% hydrogen peroxide and serum, followed by incubation with TRIM65 antibody (Sigma-Aldrich, St. Louis, MO, USA) overnight at 4°C. Slides were then incubated with goat anti-rabbit secondary antibody, developed using 3,3-diaminobenzidine (DAB) solution and counterstained with hematoxylin. The specimens were graded into three groups according to the extent of positivity as follows: Low: < 25% of the tumor cells showed positive stain; high: > 25% of tumor cells showed positive stain.

The article "Knockdown of TRIM65 inhibits lung cancer cell proliferation, migration and invasion: A therapeutic target in human lung cancer" was retracted in 2024. Reason: duplicated images.

### Silencing of TRIM65 by small interfering RNA

siRNA targeting human TRIM65 mRNA was synthesized (siRNA-TRIM65: 5’-GAUUAUCGCAAUCUGACCU-3’). A non-specific scramble siRNA sequence was used as a negative control (siRNA-NC: 5’-UUGUACUACACAAAAGUACUG-3’). The siRNA was transiently transfected into SPC-A-1 and NCI-H358 cells using Lipofectamine 2000 (Invitrogen, Carlsbad, CA, USA) according to the manufacturer's instruction. Assays were performed 48 h after transfection.

### Construction of TRIM65 stable expression vector

The TRIM65 cloning sequence was cloned into the pLV-IRES-eGFP lentiviral vector. A black pLV-IRES-eGFP lentiviral vector was used as negative control. The constructs were then transducted into HEK 293T cells with lentiviral packaging vectors by using Lipofectamine 2000 according to the manufacture's instruction. After 48 h transduction, lentivirus was collected and infected NCI-H1975 cells.

### RNA isolation and RT-PCR

Total RNAs were extracted from lung cancer tissues and cells with TRIZOL reagent (Life Technologies) according to the manufacturer's protocol. Real-time PCR (RT-PCR) was performed using SYBR Green qPCR kit (Finnzymes Oy, Espoo, Finland). GAPDH level was used as internal control and expression changes were calculated using the 2^-ΔΔCt^ method. The primers sequences (sense/antisense) used were list in Table 1.

**Table 1:** Primes sequences used in this study

Gene	Sequences
TRIM65-forward	5’-CCTTCCATGCCCTCTTCAAC-3’
TRIM65-reverse	5’-CTCCATCCCATGCCTTCTTC-3’
Bax-forward	5’-AGCTGAGCGAGTGTCTCAAG-3’
Bax -reverse	5’-TGTCCAGCCCATGATGGTTC-3’
caspase-3-forward	5’-AACTGGACTGTGGCATTGAG-3’
caspase-3-reverse	5’-ACAAAGCGACTGGATGAACC-3’
Bcl-2-forward	5’-CCACCAGCACCATAGAAG-3’
Bcl-2-reverse	5’-GAGCAGGCACAGAGAAAG-3’
Twist1-forward	5’-AGTCCGCAGTCTTACGAG-3’
Twist1-reverse MMP-2-forward	5’-GCTTGCCATCTTGGAGT-3’ 5’-TTGACGGTAAGGACGGACTC-3’
MMP-2-reverse	5’-GGCGTTCCCATACTTCACAC-3’
MMP-9-forward	5’-AAGGGCGTCGTGGTTCCAACTC-3’
MMP-9-reverse	5’-AGCATTGCCGTCCTGGGTGTAG-3’
E-cadherin-forward	5’-GAGAACGCATTGCCACATACAC-3’
E-cadherin-reverse	5’-AAGAGCACCTTCCATGACAGAC-3’
PCNA-forward	5’-GGTGTTGGAGGCACTCAAGG-3’
PCNA-reverse	5’-CAGGGTGAGCTGCACCAAAG-3’
Cyclin D1-forward	5’-AGGGAGGTGGCAAGAGTGTG-3’
Cyclin D1-reverse	5’-GCCTGGAAGTCAACGGTAGC-3’
CDC25A-forward	5’-AATACGAGGGAGGCCACATC-3’
CDC25A-reverse	5’-GACACGCTTGCCATCAGTAG-3’
KPNA2-forward	5’-AATGAGGCGTCGCAGAATAG-3’
KPNA2-reverse	5’-TTACAGTGCCCTGGTTGTTG-3’
MELK-forward	5’-ATTCTTAGGAACGCCGTACC-3’
MELK-reverse	5’-AAAGCCACCTGTCCCAATAG-3’
KIF2C-forward	5’-GGAAACGCCCACTGAATAAG-3’
KIF2C-reverse	5’-CTTGCTGTGAACCTGTAGAC-3’
RHOA-forward	5’-TCTGTCCCAACGTGCCCATC-3’
RHOA-reverse	5’-TCACCGGCTCCTGCTTCATC -3’
ROCK1-forward	5’-GTGCCACAGAGATCACTTAG-3’
ROCK1-reverse	5’-CCAGATGGTGGATTCTTAGG-3’
DLC1-forward	5’-CTTCGTGCCCTCCATGTTCC-3’
DLC1-reverse	5’-CCAGTTGCCCGTAGCCAATC-3’
ARHGAP5-forward	5’-GAAGAGACCGCCCTTACAAAGC-3’
ARHGAP5-reverse	5’-GCTCACCCGATAAATGCCATCC-3’
GAPDH-forward	5’-CACCCACTCCTCCACCTTTG-3’
GAPDH-reverse	5’-CCACCACCCTGTTGCTGTAG-3’

The article "Knockdown of TRIM65 inhibits lung cancer cell proliferation, migration and invasion: A therapeutic target in human lung cancer" was retracted in 2024. Reason: duplicated images.

### Western blot

Total proteins were isolated from cells infected with siRNA or lentivirus, and were subjected to 12% SDS-PAGE and electrophoretically transferred onto a nitrocellulose sheet. Membranes were first incubated with antibody against TRIM65, Bcl-2, Bax, caspase-3, Twist1, MMP2, MMP-9, E-cadherin, PCNA, Cyclin D1, CDC25A, KPNA2, MELK, KIF2C, RHOA, ROCK1, DLC1, ARHGAP5, P-ERK1/2, ERK1/2, P-JNK1/2, JNK1/2 and GADPH, then with anti-GAPDH antibody as an internal control. Antibodies against TRIM65, caspase-3, MMP2, MMP-9, Twist1, KPNA2, MELK, KIF2C, ROCK1, DLC1 and ARHGAP5 used in this study were purchased from Abcam (Cambridge, MA, USA). Antibodies against Bax and Bcl-2 were purchased from Santa Cruz Biotechnology (Santa Cruz, CA, USA). Antibodies against E-cadherin, PCNA, Cyclin D1, CDC25A, RHOA, P-ERK1/2, ERK1/2, P-JNK1/2, JNK1/2 and GAPDH were purchased from Cell Signaling Technology (Danvers, MA, USA). Probing and detection of specific proteins was performed with enhanced chemiluminescence (ECL, Millipore, Bredford, USA) after antibody binding. The immunoreactive bands were quantified by the densitometry with Image J software (NIH, USA).

### Cell proliferation assay

The cell proliferation was evaluated by Cell Counting Kit-8 (CCK-8) assay (Dojindo Molecular Technologies, Inc., Rockville, USA). Cells infected with siRNA or lentivirus for 48 h were plated in 96-well plates (5x10^3^ cells/well) and incubated for indicated times. After 0, 24, 48 and 72 h of incubation, CCK-8 solution (200 μl) was added to each well and incubated for an additional 1 h at 37°C. The optical density of each well at a wavelength of 450 nm was recorded on a microplate reader (Thermo Fisher Scientific, Inc.).

### Cell cycle distribution analysis

Cells infected with siRNA or lentivirus for 48 h were detached and washed with ice-cold PBS once and fixed in 70% ethanol. Fixed cells were then washed in PBS and incubated with 1 mg/ml RNase A and 0.1 mg/ml propidium iodide (PI, Sigma, St. Louis, MO, USA) for 30 min at 37°C. Intensities of fluorescence signals were measured on a flow cytometer (BD Biosciences, San Jose, CA, USA). The percentage of cells in the G0-G1, S and G2-M phases was determined using FlowJo software (version 7.6.1, Tree Star, Ashland, OR, USA).

The article "Knockdown of TRIM65 inhibits lung cancer cell proliferation, migration and invasion: A therapeutic target in human lung cancer" was retracted in 2024. Reason: duplicated images.

### Apoptosis detected by flow cytometry

Cells infected with siRNA or lentivirus for 48 h were detached and washed with ice-cold PBS. Annexin V and PI staining were carried out using the Annexin V-FITC Apoptosis Detection Kit (BD Biosciences), according to the manufacturer's instructions. After 20 min incubation in a dark at room temperature, the cells were immediately analyzed by flow cytometer.

### Cell migration and invasion assays

Cells infected with siRNA or lentivirus for 48 h were detached and washed with serum-free media. 2X10^5^ cells were resuspended in serum-free media and loaded into 8 μm membrane inserts (Corning, MA) and placed over media containing 10% fetal bovine serum. The cells migrated to the lower compartment over the time point of 24 h was scored by Toxcount (Active Motif, CA). For cell invasion assays, Matrigel (BD, CA) coating membrane inserts were used according to the manufacturer's instruction. The cells migrated to the lower compartment over the time point of 48 h was scored by Toxcount.

### Cell adhesion assay

Cells infected with siRNA or lentivirus for 48 h were seeded onto fibronectin-coated 12-well plates at a density of 1×10^5^ cells per well and allowed to adhere at 37°C for 1 h. After non-adherent cells were washed off with PBS, attached cells were fixed in 4% paraformaldehyde and stained with GIEMSA solution. The adherent cells were photographed and counted under an Olympus inverted microscope (Lake Success, NY, USA).

### *In vivo* tumorigenesis in nude mice

A total of 2 × 10^6^ logarithmically growing NCI-H358 cells with siRNA-NC or siRNA-TRIM65 infection in 0.1 ml PBS were subcutaneously injected into the right armpit of 4-week-old male BALB/c nude mice (*n* = 6) (SLAC laboratory animal Center, Shanghai, China). 45 days after injection, the nude mice were killed and tumor tissues were excised and weighed. The excised tumor tissues were formalin-fixed, paraffin-embedded, sectioned and then analyzed with Ki67 immunostaining (Abcam, Cambridge, MA, USA) or TUNEL assay (Roche Applied Science, Mannheim, Germany). All animal experiments were approved by the IACUC committee at the Northern Jiangsu People's Hospital and Clinical Medical College of Yangzhou University.

The article "Knockdown of TRIM65 inhibits lung cancer cell proliferation, migration and invasion: A therapeutic target in human lung cancer" was retracted in 2024. Reason: duplicated images.

### Gene set enrichment analysis (GSEA)

In this study, lung cancer cohort downloaded from The Cancer Genome Atlas (TCGA) was analyzed by GSEA. GSEA was performed using the GSEA software, Version 2.0.1, obtained from the Broad Institute (http://www.broad.mit.edu/gsea) as previously described [28, 29]. Gene set permutations were performed 1,000 times for each analysis. The nominal *P* value and normalized enrichment score (NES) were used to sort the pathways enriched in each phenotype.

### Co-immunoprecipitation (Co-IP)

Co-immunoprecipitation was performed as described previously [30]. Both the input and IP samples were analyzed by Western blot using various antibodies at the following dilutions: TRIM65 antibody (1:1000), RhoA antibody (1:1000), Flag-tag antibody (1:1000), HA-tag antibody (1:1000) and normal rabbit/mouse IgG (Cell Signaling Technology)

### Statistical analysis

The data was presented as the mean value ± SD. The paired, two-tailed Student's t-test and One-way analysis of variance (ANOVA) followed by Bonferroni's multiple comparison post-test were used to analyze the significance of difference between groups. Overall survival in relation to TRIM65 expression was evaluated by the Kaplan-Meyer survival curve and the log-rank nonparametric test. Differences were considered significant with a value of *P* < 0.05.

## SUPPLEMENTARY MATERIALS FIGURE


